RETRACTED

# A Green Synthesis Strategy of Binuclear Catalyst for the C-C Cross-Coupling Reactions in the Aqueous Medium: Hiyama and Suzuki–Miyaura Reactions as Case Studies

**DOI:** 10.3389/fchem.2021.747016

**Published:** 2021-11-29

**Authors:** Pouya Ghamari Kargar, Ghodsieh Bagherzade

**Affiliations:** Department of Chemistry, Faculty of Sciences, University of Birjand, Birjand, Iran

**Keywords:** ionic liquid, magnetic cellulose, cobalt, binuclear catalyst, C-C cross-coupling reactions, suzuki and hiyama-miyaura reactions

## Abstract

Cellulose, as a green and available phytochemical, was immobilized on the surface of magnetite nanoparticles then doped with imidazole and Co. complex (Fe_3_O_4_@CNF ∼ ImSBL ∼ Co.) and used as a water-dispersible, recyclable and efficient nano catalyst for the synthesis of C−C cross-coupling reactions including fluoride-free Hiyama and Suzuki reactions in an aqueous medium as an efficient and vital solvent, due to their high application and importance in various fields of science. Different spectroscopic and microscopic techniques were used for the catalyst characterization such XRD, FESEM, TEM, FT-IR, EDX, DLS, VSM, UV-Vis, and ICP analyses. The presence of imidazole as ionic section tags with hydrophilic character on the Co-complex supported on magnetic nanoparticles provides dispersion of the catalyst particles in water, which leads to both higher catalytic performance and also facile catalyst recovery and reuse six times by successive extraction and final magnetic separation. High catalytic activity was found for the catalyst and high to excellent efficiency was obtained for all Suzuki (80–98% yield; E factor: 1.1–1.9) and Hiyama (87–98% yield; E factor: 0.26–1.1) derivatives in short reaction times under mild reaction conditions in the absence of any hazardous or expensive materials. There is not any noticeable by-product found whether for Suzuki or Hiyama derivatives, which reflects the high selectivity and also the lower the E factor the more favorable is the process in view of green chemistry. The bi-aryls were achieved from the reaction of various aryl iodides/bromides and even chlorides as the highly challenging substrates, which are more available and cheaper, with triethoxyphenylsilane or phenylboronic acid. To prove the performance of the catalyst components (synergistic of SBL ∼ Co. and IL), its different homologs were incorporated individually and studied for a model reaction. Exclusively, this is an introductory statement on the use of Cobalt binuclear symmetric ionic liquid catalysts in Hiyama reactions.

## Introduction

Green chemistry is the design of chemicals and operations that minimize or remove dangerous substances from the environment. Green chemistry seeks to reduce the adverse effects of chemical experiments on the environment by preventing the contamination of resources (Kim and Li, 2020). These methods include replacing organic solvents with water, using supercritical fluids and using ionic liquids, and using non-toxic catalysts (Ran et al., 2008; Ghamari Kargar et al., 2018). It should be emphasized that these methods are complementary and in line with each other, and neither of them is superior to the other. Due to the importance of green chemistry, the principles raised in this field are discussed below. One of the essential general criteria that support chemical changes to green chemistry is low temperatures and environmentally friendly solvents and prevent the formation of waste or excess materials using heterogeneous catalysts (Zhu et al., 2010; Duan et al., 2015; Byrne et al., 2016; Ghamari Kargar et al., 2020). As an ideal renewable catalytic source, ionic liquids with non-toxic metals and magnetic substrates are the most promising options for environmentally friendly nano catalytic processes, and in general, research in the field of the nanocatalysts has always been one of the most exciting topics in nanochemistry and green chemistry (Janiak, 2013; Rathee et al., 2020).

RETRACTED

Today, nanotechnology is an influential factor in science and industry, and experts and researchers have confirmed that this technology, as an impending revolution, will seriously affect the economic future of countries and their position in the world.(de Ruiter et al., 2019). These particles have unique physical and chemical properties that are significantly different from the mass of materials. Among the types of nanoparticles, magnetic nanoparticles, owing to their simple differentiation with an exterior magnetic field and their high capacity for use in various fields from the reaction environment (Zibareva et al., 2019; Khashei Siuki et al., 2020). Magnetic nanoparticles may be slowly oxidized by surfactants, polymers, and precious metals. Therefore, to maintain the optimum properties of the nanoparticles and prevent oxidation, a stabilizer or coating must be added to protect them from wear and corrosion (Paul and Robeson, 2008; Nishino and Peijs, 2014).

In recent years, many solid substrates have been used in the construction of solid heterogeneous catalysts. One of these widely used substrates is cellulose; (Isogai et al., 2011); Nanocellulose is a unique natural substance extracted from lignocellulose materials that in the past few years owing to its remarkable physical, chemical, and biological virtues has attracted the attention of many researchers for medical and catalytic applications. In general, two types of nanocelluloses, namely cellulose nanofibers (CNF or NFC), and cellulose nanocrystals (CNC or NCC) have been introduced (Klemm et al., 2011). Cellulose nanofiber are long and flexible molecules that are about 10–100 nm thick and are composed of amorphous and crystalline parts (Isogai, 2013; Gó mez et al., 2016). In general, cellulose nanofibers by mechanical pressure and shear force and in some cases by enzymatic hydrolysis is produced. In fact, cellulose nanocrystals are rod-shaped crystals and have less flexibility than cellulose nanofibers because they lack amorphous parts (Brinchi et al., 2013; Abdul Khalil et al., 2014). Among nano cellulose, cellulose nanofibers have been extensively studied due to their excellent flexibility, biocompatibility, cheap, availability, good binding to organic molecules, thermal stability, and low toxicity, and have been considered as an option for catalytic applications (Sabaqian et al., 2017). Cellulose nanofiber (CNF) is a linear polymer with a unit glucopyranose that has biodegradable, non-toxic, recyclable, hydrophilic, and safe properties, etc., Cellulose is used in various industries like wood and paper, food industry, textile, electrical, pharmaceutical, and health, etc. (Gopiraman et al., 2018; Ghamari Kargar et al., 2020).

RETRACTED

Another important part of catalytic compounds is the presence of ionic liquids. In addition to the low vapor pressure shown by ionic liquids, these compounds can be used as recyclable catalysts due to their high ability to function as environmentally friendly alternatives to organic solvents. Without causing a reduction in its activity (Plechkova and Seddon, 2008; Sowmiah et al., 2009). Also, ionic liquids have other interesting virtues like thermal and chemical fixity, great ionic conductivity, and a wide range of electrochemical potentials. Recent activity in ionic liquids has shown that these compounds can be used as catalysts and solvents in organic reactions (Kaur, 2018). Water, for reasons such as non-flammability, non-toxicity, great dielectric constant, and environmental friendliness, is the best candidate as a solvent in organic syntheses and mating reactions. The formation of new carbon-carbon bonds in organic chemistry is so important that these reactions are considered a prerequisite for life on Earth. Carbon-carbon coupling reactions come in many forms, some of the most important of which are discussed, including Hiyama and Suzuki–Miyaura (Veisi et al., 2017; Marset et al., 2018; Monfared et al., 2019). These reactions were performed with the help of intermediate metal complexes as catalysts. They enabled the formation of carbon-carbon bonds for substrates with sensitive functional groups. They were quickly able to find many applications in various scientific fields, including biochemistry, process chemistry, pharmaceutical chemistry, and nanotechnology (Bedford, 2003), (Szabó, 2006; Johansson Seechurn et al., 2012). Among the transition metals, palladium was selected as catalyst for Hiyama and Suzuki-Miyaura cross-coupling reactions. It is still considered the most popular metal for C-C bonding reactions.

RETRACTED

Despite these advantages, the Hiyama and Suzuki couplings are usually performed in common organic solvents and expensive catalysts, which usually have high toxicity, flammability, and vapor pressure even at low temperatures resulting in serious environmental concerns. As reported by U.S. FDA guidelines (CDER 2017), the commonly used solvents for the Hiyama reactions such as tetrahydrofuran (Miller and Montgomery 2014) dioxane (Zhang et al., 2014), N, N-dimethylfor-mamide (Handy et al., 2005), toluene (Denmark et al., 2010), and 1,2-dichloroethane (Ramgren and Garg 2014) are classified into Class 1 and 2, which utilizations should be avoided or limited, respectively, particularly in the pharmaceutical industry. To eliminate these hazardous auxiliary materials, the reactions have been demonstrated in alternative media, e.g., water (Sakon et al., 2017) or glycerol (Marset et al., 2018). Although, numerous Pd-catalyzed coupling Suzuki reactions like FS-PdCl_2_, (Yang et al., 2021), boehmite@tryptophan-Pd, (Ghorbani et al., 2019), L-methionine-Pd, (Mohammadi et al., 2020), Pd@NC NPs, (Aabaka et al., 2021), Fe_3_O_4_–Pd-biochar, (Akay et al., 2021), [Pd (bzq) (μ-Cl)]2, (Samiee et al., 2021), were demonstrated. However, palladium complexes have restrictions such as high toxicity, cost, renewable, and sensibility to air (Loska et al., 2008; Jismy et al., 2021). Thus, the development of a simple, convenient, and environmentally benign method for synthesizing Suzuki and Hiyama remains necessary. Also, by the introduction of a biomass-based solvent into this synthetically important reaction, the environmental impacts of a Hiyama and Suzuki reactions involved synthesis could be further controlled and reduced. However, to achieve good results in the reaction process, it is crucial to choose a suitable heterogeneous catalyst and an environmentally benign method that can overcome all these problems. For minimizing chemical waste, increasing energy efficiency, and obtaining better economy, the use of nanocatalysts that comply with the principles of green chemistry is recommended.

However, cobalt catalysts are important because of their low cost, non-toxicity, and availability. The use of this metal catalyst in coupling reactions is rare to resemble the previously mentioned metal catalysts in the article. However, cross-coupling reactions catalyzed by transporting metals are the most common, most straightforward, and most impressive conventions for preparing C-C bonds in organic chemistry. Meanwhile, the Hiyama and Suzuki-Miyaura cross-coupling reactions have engrossed considerable consideration for the efficacious and straightforward synthesis of biaryls from aryl halide reactions and organosilicon/organoboron reagents. Inspired by this verity and as a section of our ongoing efforts to develop new catalytic methods to perform cross-coupling reactions through more benign environmental conditions, here, we have successfully introduced binucler catalyst on the magnetic cellulose nanofiber with Schiff base Co. (denoted as Fe_3_O_4_@CNF ∼ ImSBL ∼ Co.). We have synthesized it as a separable cobalt dual-core magnetic nanocatalyst and evaluated it by various techniques. The nanocatalyst capability has been well investigated due to the Hiyama and Suzuki-Miyaura junction interactions at 70 and 80^o^C in an aqueous medium (Scheme 1).

RETRACTED

**SCHEME 1:** The catalytic activity of the Fe_3_O_4_@CNF ∼ ImSBL ∼ Co. nanocatalyst Hiyama and Suzuki–Miyaura cross-coupling reactions.

## Materials and Methods

### Chemicals and Physicochemical Characterization

The catalyst was characterized by several techniques, including ICP, XRD, EDX, FT-IR, TEM, Fe-SEM, DLS, and VSM. All chemicals were purchased from Sigma and Merck and used without any further purification. All solvents were distilled and dried before use. The progress of the reactions and the purity of the products were determined by TLC on silica-gel Polygram SILG/UV254 plates. Fourier transform infrared (FT-IR) spectra were recorded with a Nicolet system 800 beam splitter KBr SCAL = 800 in the range 400–4,000 cm^−1^. The resolution of FT-IR analysis and the number of scans for each sample were 4 cm^−1^ and 16 times, respectively. The FT-IR measurement is a reliable technique for a quantitative measurement of catalyst and used a room temperature detector. NMR spectra were recorded in DMSO-d6 using a Bruker Advance DPX-400 and 250 instruments using tetramethylsilane as internal standard. The powder X-ray diffraction pattern of Fe_3_O_4_@CNF ∼ ImSBL ∼ Co. was obtained with an X'Pert Pro MPD diffractometer with a Cu Kα (*λ* = 1.54060 Å). All powder samples were recorded from Bragg angle, 2θ of 10°–80° at scan speed = 1 min^−1^ and step size = 0.05°. Transmission electron microscopy (TEM) images were obtained using a Philips CM120 microscope. ICP analysis was performed by VARIAN VISTA-PRO CCD simultaneous ICP-OES instrument. The elements in the samples were probed by energy-dispersive X-ray (EDX) spectroscopy accessory to the Philips scanning electron microscopy (SEM). The magnetization behaviour of the NPs was investigated on a Lake Shore vibrating sample magnetometer (VSM) at room temperature. The Zeta-potential is determined by zeta potential analyzer and hydrodynamic diameter is determined by DLS (dynamic light scattering) on a HORIBA-LB550 instrument.

RETRACTED

### Preparation of Fe_3_O_4_ and Fe_3_O_4_@CNF Core-Shell NPs (1)

Magnetic nanoparticles Fe_3_O_4_ and core-shell Fe_3_O_4_@CNF nanospheres were prepared according to a previously mentioned (Scheme 2; Ghamari Kargar et al., 2020).

**SCHEME 2:** Hyiama reaction of aryl halides with triethoxyphenylsilane catalyzed by Fe_3_O_4_@CNF ∼ ImSBL ∼ Co. in water.

### Approach for the Synthesis of Imidazole Moiety Based on Fe_3_O_4_@CNF_∼_CPTMS (Fe_3_O_4_@CNF_∼_Im) (2)

In the first step, imidazole (5 mmol, 0.34 g) was dissolved in (5 ml) of dry toluene, and then 3-chloropropyl-trimethoxy silane (CPTMS: 5 mmol, 0.9 ml) was added slowly to the mixture. The mixture was then stirred for 3 h at room temperature. After stirring, the product obtained from imidazole and CPTMS was gently added for 30 min to Fe_3_O_4_@CNF (1.5 g) stirred in dry toluene solution (30 ml) while sonicating. The reaction was exposed for 24 h under N_2_ gas at reflux conditions. Then the flask content was stirred with Et_3_N (0.5 ml) for 30 min at room temperature. After finishing the reaction, the solid obtained is separated by an exterior magnet and washed with toluene and diethyl ether. At the end, solid dried in a vacuum oven at 70°C for 24 h.

### Synthesis of Schiff Base Ligand (SBL) (3)

In the beginning, 2-hydroxy-5-chloromethyl benzaldehyde was synthesized and purified under a previously illustrated procedure (Ghamari kargar et al., 2021) (purple solid, 98% yield, mp: 86–87^o^C). 2-Hydroxy-5- chloromethyl benzaldehyde (2.0 mmol, 0.34 g) was dissolved in 10 ml of CH_2_Cl_2,_ and then p-Phenylenediamine (1.0 mmol, 0.108 g) was added to the mixture. The contents of the flask were stirred for 4 h at boiling temperature. After reflux, in order to separate the solvent from the obtained precipitate, the desired product Schiff base ligand 6,6'-((1E,1′E)-(1,4-phenylene bis (azaneylylidene)) bis(methaneylylidene)) bis(3-(chloromethyl) phenol) (SBL: IV) was centrifuged and washed with cold CH_2_Cl_2_ and diethyl ether and dried at ambient temperature (Supporting information, Scheme 2). Spectral information of 2-hydroxy-5-chloromethyl benzaldehyde composition:

FT-IR (KBr): = 3,151 (O-H), 3,033, 2,975, 2,865 (C-H aldehyde), 1,665 (C=O), 1,434 (C=C), 673 (CH_2_-Cl) cm^−1^.

^1^HNMR (DMSO, 300 MHz): *δ* = 4.80 (s, 2H, CH_2_), 7.56–7.60 (d,d, 2H, H-Ar), 7.72 (s, 1H, H-Ar), 10.06 (s, 1H, CH of aldehyde), 11.30 (s, 1H, O-H) ppm.

^13^CNMR (DMSO, 75 MHz): *δ* = 47.0, 117.8, 124.8, 131.1, 136.1, 136.4, 148.4, 163.2, 197.7 ppm.

RETRACTED

Spectral information of 6,6'-((1E,1′E)-(1,4-phenylenebis (azaneylylidene)) bis(methaneylylidene)) bis(3-(chloromethyl) phenol) composition:

^1^HNMR (DMSO, 300 MHz): *δ* = 4.27 (s, 4H, CH_2_-Cl), 6.74 (s, 4H, H-Ar), 6.94 (s, 2H, H-Ar), 7.13–7.15 (d, 2H, H-Ar), 7.91–7.93 (s, 2H, H-Ar), 8.72 (s, 2H, CH = N), 9.94 (s, 2H, O-H) ppm.

^13^CNMR (DMSO, 75 MHz): *δ* = 56.4, 111.9, 116.2, 123.5, 129.5, 134.7, 146.7, 159.2, 162.8 ppm.

### Synthesis of Complex SBL by Co.(OAc)_2_ (4)

After the formation of the desired ligand (V), the next step was dissolving of Co(OAc)_2_ (10 M) in EtOH (25 ml) by stirring at room temperature. Then SBL (1 mmol) was sonicated with a minimum volume of EtOH and added the above solution under stirring. The solid was filtered off, washed with EtOH and finally with diethyl ether and dried in vacuo.

### Approach for the Synthesis of SBL _∼_ Co. Based on Fe_3_O_4_@CNF ∼ Im (Fe_3_O_4_@CNF ∼ ImSBL ∼ Co.) (5)

The synthesized Fe_3_O_4_@CNF ∼ Im (1.5 g) was added to a flask containing 15 ml of dry toluene in a sonicate for 15 min. The solvent suitable for this stage of the reaction is dry toluene, which SBL ∼ Co. (5 mmol) was dissolved in dry toluene (20 ml) added dropwise to the dispersed mixture and stirred at 75^o^C for 24 h. The solid obtained was separated by an exterior magnet and was washed with toluene and diethyl ether. In the end, we dried the solid in a vacuum oven at 70°C for 24 h.

#### A General Approach for Hiyama Cross-Coupling Reaction

A mixture of Fe_3_O_4_@CNF ∼ ImSBL ∼ Co. (0.3 mol%) in 3 ml of H_2_O was stirred for 5 min. Then, in a typical run, aryl halide (1.0 mmol) and NaOH (2 mmol), and triethoxyphenylsilane (1.5 mmol) were added, and the resultant mixture was stirred at 70^o^C in an oil bath. The reaction progress was monitored by TLC. After completion of the reaction, the reaction mixture cooled to room temperature. The organic layer was extracted with CH_2_Cl_2_ (2 × 10 ml) from the aqueous layer. Using anhydrous Mgso_4_ organic layer was dried, filtered, and the solvent was removed under reduced pressure. The catalyst has remained in the aqueous layer for reuse.

#### A General Method for Suzuki–Miyaura Cross-Coupling Reaction

A mixture of Fe_3_O_4_@CNF ∼ ImSBL ∼ Co. (0.3 mol%) in 3 ml of H_2_O was stirred for 5 min. Then, in a typical run, aryl halide (1.0 mmol) and K_2_CO_3_ (2 mmol), and phenylboronic acid (1 mmol) were added, and the resultant mixture was stirred at 70°C in an oil bath. The reaction progress was monitored by TLC. After the reaction is completed, allowed the mixture to cool. The organic layer was extracted with CH_2_Cl_2_ (2 × 10 ml) and dried by anhydrous MgSO_4_. Then the solvent under reduced pressure was removed. The catalyst is in the aqueous phase and will be separated for another run.

RETRACTED

#### Spectral Data

##### 1,1′-Biphenyl

^1^HNMR (DMSO-d_6_, 400 MHz): *δ* = 7.52–7.47 (t, 2H, j = 20 Hz), 7.67–7.62 (t, 4H, j = 20 Hz), 7.91–7.88 (t, 4H, j = 12 Hz) ppm.

^13^CNMR (DMSO-d_6_, 100 MHz): *δ* = 128.3, 128.4, 129.3, 141.8 ppm.

##### 4-Nitro-1.1′-Biphenyl

^1^HNMR (DMSO-d_6_, 400 MHz): *δ* = 7.35–7.40 (t, 1H, j = 20 Hz), 7.47–7.52 (t, 2H, j = 20 Hz), 7.89–7.92 (d, 2H, j = 12 Hz), 8.32–8.37 (d, 2H, j = 20 Hz), 8.43–8.48 (d, 2H, j = 20 Hz) ppm.

^13^CNMR (DMSO-d_6_, 100 MHz): *δ* = 125.61, 127.4, 127.7, 129.8, 130.2, 140.5, 146.7, 146.8 ppm.

##### 4-Methoxy-1,1′-Biphenyl

^1^HNMR (DMSO-d_6_, 400 MHz): *δ* = 4.01 (s, 3H, CH_3_), 7.07–7.09 (d, 2H, j = 8 Hz), 7.37–7.3 (m, 3H), 7.47–7.49 (d, 2H, j = 8 Hz) ppm.

^13^CNMR (DMSO-d_6_, 100 MHz): *δ* = 55.3, 114.2, 127.4, 127.7, 129.3, 131.1, 133.4, 141.8 ppm.

##### 4-Chloro-1,1′-Biphenyl

^1^HNMR (DMSO-d_6_, 400 MHz): *δ* = 7.34–7.39 (t, 1H, j = 20 Hz), 7.46–7.51 (t, 2H, j = 20 Hz), 7.84–7.86 (d, 2H, j = 8 Hz), 7.89–7.91 (d, 2H, j = 8 Hz), 8.03–8.07 (d, 2H, j = 16 Hz) ppm.

^13^CNMR (DMSO-d_6_, 100 MHz): *δ* = 127.7, 128.0, 129.1, 129.3, 133.4, 138.2, 140.1 ppm.

##### [1,1′-Biphenyl]-4-Carbonitrile

^1^HNMR (DMSO-d_6_, 400 MHz): *δ* = 7.07–7.09 (d, 2H, j = 8 Hz), 7.37–7.45 (m, 3H), 7.83–7.87 (d, 2H, j = 16 Hz), 7.96 (s, 4H) ppm.

^13^CNMR (DMSO-d_6_, 100 MHz): *δ* = 111.9, 118.1, 127.5, 127.7, 127.8, 129.8, 133.4, 140.2, 144.4 ppm.

## Results and Discussion

Green chemistry, also called sustainable chemistry, is a research philosophy in chemistry that aims to design products and processes, including environmentally friendly catalysts. Also, The ionic liquid section of special importance in green chemistry. Green chemistry seeks to reduce and prevent environmental pollution, As the importance of green chemistry has increased during the last decade, therefore synthesizing new recyclable nano catalyst has been a focus of the scientific community. In order to study the catalysts, a heterogeneous, magnetically recoverable Fe_3_O_4_@CNF ∼ ImSBL ∼ Co. nano catalyst was prepared by immobilization of a novel Co. (II) Schiff base complex on Fe_3_O_4_@CNF nanoparticles followed by treatment with imidazole, and was found to be an efficient catalyst for the Suzuki and Hiyama reactions. This catalyst can be a suitable option for organic syntheses as it has features such as simple synthesizing and recovery, non-toxicity, and high catalytic output.

RETRACTED

## Catalyst Characterization

In this work, FT-IR spectra of the compounds 1, 2, 3, 4, 5 are shown in Figures 1A–G. As is clear in Figure 1A, the characteristic peaks at 731 cm^−1^ (C–Cl stretching vibration), 1,107 cm^−1^ (C–O stretching vibration), 1,450–1,580 cm^−1^ (C=C aromatic stretching vibration), 1,652 cm^−1^ (C=O stretching vibration), and 2,809 cm^−1^ (C–H aldehyde stretching vibration), 2,980 cm^−1^ and 3,100 cm^−1^ (C–H aliphatic and aromatic stretching vibration), 3,250 cm^−1^ (O–H stretching) supports the structure of 2-hydroxy-5-chloromethyl benzaldehyde (Figure 1A). FT-IR spectrum of compound 3 (Figure 1B), illustrates the Schiff base reaction between *p*-phenylendiamine and 5-chlorosalicylaldehyde, the characteristic peaks at 745 cm^−1^ (C–Cl stretching), 1,520 cm^−1^ (C=C aromatic stretching vibration), 1,643 cm^−1^ (C=N stretching vibration) 2,965–3,080 cm^−1^ (C–H aliphatic and aromatic stretching vibration), and 3,400 cm^−1^ (O–H stretching) supports the structure of SBL. Figure 1C, signs the FT-IR spectrum of Fe_3_O_4_ nanoparticles with two characteristic peaks at 3,402 cm^−1^ and 578 cm^−1^ related to O–H and Fe–O stretching bands, sequentially, that confirms the formation of Fe_3_O_4_ nanoparticles. In addition to the peak Fe-O, the strong peak at 3,300 cm^−1^ shows the (O–H stretching vibrations) of cellulose nanofibers (Figure 1D). Non-overlapping characteristic absorbance peaks for the reaction between CPTES and imidazole allow fast and reliable KBr-FTIR quantitative measurements to distinguish among major component groups. FTIR spectrum of compound PTMS-Im exhibits the absorption bands at 1,100–1,200 cm^−1^ (C–O, C-N, Si-O stretch), 1,475–1,590 cm^−1^ (Aromatic Str. C=C), 1,648 cm^−1^ (C=N stretch), and 2,989 cm^−1^ (C-H stretching) (Figure 1E). These absorption peaks confirm the successful preparation of PTMS-IM. Figure 1F shows the FT-IR spectrum strong peak of Si–O and C-N stretching vibration at 1,020–1,110 cm^−1^ and 3,120 cm^−1^ C–H aromatic stretching vibration referring to the imidazolium linkage peak to the aromatic ring (Fe_3_O_4_@CNF ∼ Im). These absorption peaks confirm the successful preparation of the catalyst. Complexation of cobalt ions to ligand SBL causes the imine peak absorption (1,643 cm^−1^) to lower wavenumbers (1,623 cm^−1^) by about 20 cm^−1^, indicating the participation of azomethine nitrogen in bonding with metal ion and supporting the coordination of stretch to the metal *via* a nitrogen atom (Figure 1G). The main absorption bands at 570 cm^−1^ (Fe–O), 1,015 cm^−1^ (Si–O), 1,490 cm^−1^ (C=C), 1,623 cm^−1^ (C=N) in the FT-IR spectrum of Fe_3_O_4_@CNF ∼ ImSBL ∼ Co., represent the functionalization of Fe_3_O_4_@CNF nanoparticles with Co. (II) complex 5 (Figure 1G).

RETRACTED

**FIGURE 1:** FT-IR spectra of **(A)** 2-hydroxy-5-chloromethyl benzaldehyde, **(B)** SBL, **(C)** Fe_3_O_4_, **(D)** Fe_3_O_4_@CNF, **(E)** PTMS-Im, **(F)** Fe_3_O_4_@CNF ∼ Im, **(G)** Fe_3_O_4_@CNF ∼ ImSBL ∼ Co.

The size and morphology of the nanoparticles were observed using transmission electron microscopy (TEM). TEM images show that the particle size has changed after immobilization of complex on modified MNPs (Figure 2). The synthesized catalysts are well dispersed and most of the nanoparticles are almost spherical in shape. The average particle size estimated about 25 nm for Fe_3_O_4_@CNF ∼ ImSBL ∼ Co. (Figure 3).

**FIGURE 2:** TEM images of Fe_3_O_4_@CNF ∼ ImSBL ∼ Co.

**FIGURE 3:** Particle size distribution histogram of Fe_3_O_4_@CNF ∼ ImSBL ∼ Co.

Since the cobalt and Fe_3_O_4_ is paramagnetic in nature the NMR technique was not performed (Shaygan et al., 2018) Therefore the presence of C, N, O, Si, Fe and Co. was detected by X-ray scattering (EDS) scattering analysis (Figure 4), which confirms the synthesis steps of the catalyst and proposed formula Fe_3_O_4_, Fe_3_O_4_@CNF ∼ Im, SBL ∼ Co., Fe_3_O_4_@CNF ∼ ImSBL ∼ Co. with quantitative measurements.

**FIGURE 4:** EDS analysis of **(A)** Fe_3_O_4_@CNF ∼ ImSBL ∼ Co., **(B)** Fe_3_O_4_, **(C)** Fe_3_O_4_@CNF ∼ Im, **(D)** SBL ∼ Co.

The vibrating sample magnetometry (VSM) analysis results for Fe_3_O_4_, Fe_3_O_4_@CNF, and Fe_3_O_4_@CNF ∼ ImSBL ∼ Co. complex nanocomposites are shown in Figure 6A. The nanoparticles exhibited high penetrance under magnetization, which was adequate to entirely separate it from an external magnet. Magnetic measurements illustrated satiation magnetization values of 63.93, 53.91, and 51.90 emu. g^−1^, respectively for Fe_3_O_4_, Fe_3_O_4_@CNF, and Fe_3_O_4_@CNF ∼ ImSBL ∼ Co. complex nanocomposites (Figure 5B). These results illustrate that the magnetization of Fe_3_O_4_ reduced extremely due to the attendance of coated Nanofiber cellulose shell and Co-Schiff base complex on its surface (Figures 5B,C). Nevertheless, the Fe_3_O_4_@CNF ∼ ImSBL ∼ Co. nanocatalyst exhibits super magnetic properties and high magnetic values that allow it to be easily separated from the mixture with a simple external magnet.

**FIGURE 5:** VSM pattern **(A)** Fe_3_O_4_, **(B)** Fe_3_O_4_@CNF and **(C)** Fe_3_O_4_@CNF ∼ ImSBL ∼ Co.

The TGA analysis was behavior to determine the uncoated Fe_3_O_4_ NPs, and content in the Fe_3_O_4_@CNF ∼ ImSBL ∼ Co. nanocatalyst. The results are illustrated in Figure 6. The TGA analysis was accomplished to confirm the coating of organic content on the surface of the Fe_3_O_4_ NPs. TGA spectra of uncoated Fe_3_O_4_ NPs show little weight loss, which is about 10% in the range of 25–800°C. This might be due to the loss of residual water in the uncoated Fe_3_O_4_ NPs (Ghamari kargar et al., 2021). Comparing with the catalyst curve, Figure 6 illustrates the thermal decomposition diagram for Fe_3_O_4_@CNF ∼ ImSBL ∼ Co. synthesized by the green method. The first mass reduction phase occurred at 25–125°C, caused by the water’s loss absorbed in the nanocatalyst surface. The second phase occurred at 150–350°C, which could have arisen due to the breakdown of the bonds and destruction of the cellulose structure (Kumawat et al., 2017). The third stage of the weight loss in the temperature range between 350 and 550°C may be due to the thermal crystal phase alteration from Fe_3_O_4_ to *?*-Fe_2_O_3_ (Ghamari Kargar et al., 2020). Other stages of weight loss up to 800°C may be due to the decomposition of organic moieties on the surface of the Fe_3_O_4_@CNF core–shell nanoparticles.

RETRACTED

**FIGURE 6:** TGA curves for **(black line)** Fe_3_O_4_, and **(yellow line)** Fe_3_O_4_@CNF ∼ ImSBL ∼ Co.

As shown in Figure 7, the X-ray diffraction pattern of crystalline structures of Fe_3_O_4_ NPs and core–shell magnetic Fe_3_O_4_@CNF ∼ ImSBL ∼ Co. show characteristic diffraction peaks correspond to (220), (311), (400), (422), (511) and (440) reflections of inverse spinel Fe_3_O_4_ NPs, respectively. It showed characteristic peaks, and the relative intensity matched well with those of standard Fe_3_O_4_ nanoparticles (reference JCPDS card no. 87–2,334) (see Figure 7) (Ghamari kargar et al., 2020). The XRD pattern Cobalt matches well with the characteristic peaks of naked Fe_3_O_4_, which illustrates maintenance of the crystalline spinel ferrite core structure during functionalization of magnetic nanoparticles. Strong peaks at 2θ = 19.91°, 30.4°, 36.3°, 54.1°, 57.7°, 63.2°, 69.9°, and 73.5° corresponding to the (001), (100), (011), (012), (110), (111), (103), and (201) crystallographic phases in XRD pattern are related to Co(OAc)_2_. (Cheng et al., 2012). The week broad peak appeared in the range from 2θ = 17.9–20.1 indicates the existence of amorphous cellulose. The crystal size of Fe_3_O_4_ NPs and core–shell magnetic Fe_3_O_4_@CNF ∼ ImSBL ∼ Co. were determined by using the Debye–Scherrer (d_{hkl}_ = 0.94 *λ*/βcosθ) equation where *ß* is the half-width of the highest intensity X-ray diffraction lines, d is the average crystalline diameter, 0.94 is the Scherrer constant, *?* is the Bragg angle in degree and *?* is the X-ray wavelength. Here, the (311) peak of the highest intensity was selected and d_311_ obtained 25 nm for Fe_3_O_4_ NPs. Comparing between X-ray diffraction pattern of Fe_3_O_4_ NPs and Fe_3_O_4_@CNF ∼ ImSBL ∼ Co. shows that the coating of cellulose and SBL ∼ Co. complex on Fe_3_O_4_ NPs did not significantly affect the structure of NPs.

RETRACTED

**FIGURE 7:** XRD spectra of **(A)** Co(OAc)_2_, **(B)** Fe_3_O_4_, **(C)** Fe_3_O_4_@CNF ∼ ImSBL ∼ Co.

Electronic spectrum of Co.(OAc)_2_, Fe_3_O_4_, Fe_3_O_4_@CNF, and Fe_3_O_4_@CNF ∼ ImSBL ∼ Co. were carried out in H_2_O as a solvent at the region of 200–800 nm (Figure 8). The synthesized Fe_3_O_4_ shows the maximum absorption peak at 360 nm. The spectrum of aqueous Fe_3_O_4_@cellulose solution exhibited a maximum at 250 and 275 nm, which was attributed to the absorption of cellulose in Fe_3_O_4_ NPs structure, which is masked after immobilization of Schiff base nickel complex by *p*-π* absorptions. In the UV-Vis spectrum the catalyst lmax and adsorption intensity appear in 355 nm, while the Co(OAc)_2_ lmax is in region 500 nm, resulting in UV-Vis spectrum of Schiff base ligand to Co(II) caused the reduction of absorption intensity of n–π* for C=N bond and π–π* transitions for benzene ring, which confirmed the successful chelation of Co(II) to the catalyst. Furthermore, the absence of resonant peak above 450 nm proved the metallic nature of Fe_3_O_4_@CNF NPs (Figure 8). According to the Tanabe-Sugano diagram in case Fe_3_O_4_, we expect a transition from T2g to eg. This transition should be slightly shoulder due to the effect of Yan Teller, which can be seen in the spectrum. However, after binding to cellulose and cobalt complex, this peak has shifted, which indicates the confirmation of cellulose adsorption to nanoparticles as well as cobalt complex (stronger ligand field and therefore more fission of d orbitals and thus shift to wavelength Shorter).

**FIGURE 8:** UV-Vis spectra of Co(OAc)_2_, Fe_3_O_4_, Fe_3_O_4_@CNF, and Fe_3_O_4_@CNF ∼ ImSBL ∼ Co. in H_2_O solvent.

FE-SEM images were used for further research of the surface morphology of the prepared catalyst. FE-SEM analysis was performed for successive synchronization stages of catalyst (Figures 9A–D). According to FE-SEM images, the synthesized Fe_3_O_4_ and Fe_3_O_4_@CNF are approximately spherical and well dispersed, albeit in some area’s larger structures with non-spherical morphology are perceived (Figures 9A,C). The SEM images also confirm the spherical structure of the Fe_3_O_4_ and show that the Fe_3_O_4_ have a homogeneous distribution and are uniform in size in accordance with the TEM image. The FE-SEM images show an increase in the size of the Fe_3_O_4_ at each step, in accommodation with the DLS results. It is interesting that the resulting spherical morphology of Fe_3_O_4_@CNF and catalyst 8 shows that the functionalization of the NPs by the silica and cobalt complexes, respectively, was accomplished regularly, and harmoniously, with no aberration in shape or aggregation in the particles. The Fe_3_O_4_ and Fe_3_O_4_@CNF particles have an average diameter of 13–15 and 20–22 nm (Figures 9A,C), respectively, consistent with their corresponding DLS analyses (Figures 9B, D). As shown in Figure 9E, FE-SEM image, clearly show a combination of organic and inorganic different components in a homogeneous network of Fe_3_O_4_@CNF ∼ ImSBL ∼ Co. 9), which has an average diameter of 35–43 nm (Figure 9F). Besides, the best technique for verification of catalyst preparation incredibly problematic half, is inductively coupled plasma optical emission spectroscopy (ICP-OES) analysis. Loading amount of Co. on the catalyst was measured by inductively coupled plasma optical emission spectroscopy (ICP-OES) instruments due to more ensure attainment. The experiment indicated that 1.5 mmol of Co. metal per Gram of the catalyst was loaded on the catalyst framework Fe_3_O_4_@CNF ∼ ImSBL ∼ Co. Also, the analyses give the percentage of the heavy metals as: 46.42 %w, 2.25 %w, 7.9 %w for Fe, Si, Co. respectively.

RETRACTED

**FIGURE 9:** Field emission-scanning electron microscopy images and dynamic light scattering results of **(A, B)** Fe_3_O_4_, **(C, D)** Fe_3_O_4_@CNF, and **(E, F)** Fe_3_O_4_@CNF ∼ ImSBL ∼ Co. complex nanocomposite.

In order to further prove the influence of cellulose polymer and organic compounds (Im, SBL-Co) on the property of Fe_3_O_4_ nanoparticles, zeta potentials of bare Fe_3_O_4_, Fe_3_O_4_@CNF and Fe_3_O_4_@CNF ∼ ImSBL ∼ Co. were collected at different pH values. The zeta potentials, as a measurement of repulsive or attractive forces between particles, play an important role to find not only the isoelectric point (pI), but also the colloidal dispersion stability. The distinct surface composition of the coated particles was further confirmed by differences in the surface charge of the nanoparticles (Figure 10). The surface charge was assessed by zeta potential (*ζ*) measurements at variable pH. Bare magnetic nanoparticles (Fe_3_O_4_) present an isoelectric point (IEP) at ca. 4.5 that is relatively below the usual IEP values reported for magnetite and can indicate oxidation of the particles surface. (Plaza, R.C et al., 2002). Nevertheless, the IEP value here obtained is in agreement with values reported for bare Fe_3_O_4_ nanoparticles prepared by oxidative hydrolysis. (Riggio, C et al., 2012). At lower pH values the surface is positively charged while at higher pH values the overall charge of the surface is negative. The isoelectric point shifts to high values in the nanoparticles coated with cellulose shells of CNF ( ∼ 5). This shift can be ascribed to hydroxyl groups present on particles surface cellulose. The zeta potential value of Fe_3_O_4_@CNF ∼ ImSBL ∼ Co. switched to a positive value after being modified with imidazole and SBL ∼ Co., indicating that imidazole and SBL ∼ Co. molecules were coated on the surface of Fe_3_O_4_@CNF. The measured potential value for Fe_3_O_4_@CNF ∼ ImSBL ∼ Co. was -20.0 mV.

RETRACTED

**FIGURE 10:** Zeta potential values of bare magnetite and coated particles at variable pH.

The specific surface area and porosity of the samples were investigated by N_2_ adsorption–desorption isotherm analysis. The specific surface area values, the average pore diameter (according to the BJH method), and the total pore volume are tabulated in Table 1. According to the BET isotherm, the active surface area of Fe_3_O_4_, Fe_3_O_4_@CNF, Fe_3_O_4_@CNF ∼ Cl, Fe_3_O_4_@CNF ∼ Im, and the Fe_3_O_4_@CNF ∼ ImSBL ∼ Co. nano catalyst were determined as 480, 460, 415, 400, and 365 m^2^ g^−1^, respectively (Table 1, entries 1–4). According to the results, the specific surface area decreased after intercalation of the melamine. However, on the other hand, the pore volume and average pore radius increased when melamine was added. These results quantitative measurements propose that the intercalation of melamine leads to the formation of a more porous network structure.

**TABLE 1:** Surface characteristics of Fe_3_O_4_, the Fe_3_O_4_@CNF, Fe_3_O_4_@CNF ∼ Cl, Fe_3_O_4_@CNF ∼ Im, and the Fe_3_O_4_@CNF ∼ ImSBL ∼ Co.

Entry	Sample	Specific surface area (m^2^.g^−1)^	Pore volume (cm^3^.g^−1^)	Average pore radius (nm)
1	Fe_3_O_4_	480	0.803	1.254
2	Fe_3_O_4_@CNF	460	0.790	1.795
3	Fe_3_O_4_@CNF ∼ Cl	415	0.755	1.805
4	Fe_3_O_4_@CNF ∼ Im	400	0.705	1.815
5	Fe_3_O_4_@CNF ∼ ImSBL ∼ Co.	365	0.730	1.825

### Optimization of the C-C Cross-Coupling Reaction Conditions Using Fe _3_O_4_@CNF_∼_ImSBL_∼_Co.

After successful characterization of the synthezed Fe_3_O_4_@CNF ∼ ImSBL ∼ Co., its catalytic activity was evaluated in C-C cross coupling reactions including Hiyama and Suzuki–Miyaura. An efficacious technique for detecting the optimum conditions in organic reactions is the statistic method reply that chemists enable to study the influx of parameter factors each other in the minim time. For more information on the cross-coupling reactive conditions, four functional parameters including solvent, temperature, base, and amount of catalyst in different conditions were examined for Hiyama and Suzuki–Miyaura cross-coupling reactions, which are efficient and useful tools in organic chemistry for synthesis. Our research on the advancement of novel catalytic systems to accomplish cross-coupling reactions by environmentally friendly methods. Here, we investigate the catalytic activity of Fe_3_O_4_@CNF ∼ ImSBL ∼ Co. in Hiyama cross-coupling reactions in the presence of an aqueous solvent. According to our literature review, this catalyst may be one of the first reports of using an ionic liquid catalyst in the presence of cobalt metal in the Hiyama cross-coupling reaction. Initially, the catalytic properties of Fe_3_O_4_@CNF ∼ ImSBL ∼ Co. were examined in Hiyama reaction. In order to find the best conditions for Hiyama reaction, the coupling of iodobenzene (1 mmol) with triethoxyphenylsilane (1.5 mmol) under different conditions was selected as the model reaction. Selected optimization range achieved for Hiyama cross-coupling reaction including nine solvents, in the presence of four bases, and 0.1–0.4 mol% amount of catalyst, and at 70–98°C. Hence, in general, the optimal points for the Hiyama reaction were investigated. Introductory results demonstrated the maximum yields in water as a green solvent for all two reactions due to the high dispersion of catalyst and strong interaction of active sites with the reactants in this medium (Table 2, entry 4). Various parameters of the reaction, including temperature, base, and amount of catalyst were evaluated for the reaction model (Hiyama), and the results are summarized in a table 2. As shown in table 2, water as a solvent showed a higher efficiency compared to all solvents tested with 98% isolated yield. To show the effectiveness of water in the reaction, some experiments were performed on an aqueous organic solvent mixture. As shown in table 2, NaOH is the most effective base for this adsorption, probably due to its good solubility in water compared to other bases (Entry 10–12). Different amounts of catalyst were investigated in Hiyama reactions. As shown in Table 2, entry 13–16, by increasing the value catalyst to 0.4 mol%, the efficiency increases linearly to 98%. Increasing the amount of catalyst by more than 0.3 mol% does not affect the efficiency percentage.

RETRACTED

**TABLE 2:** Optimization of the reaction conditions for the C-C cross coupling of iodobenzene with triethoxyphenylsilane.

Entry	Solvent	Base	Catalyst (mol%)	Temp. (^o^C)	Time (h)	Yield^a^ (%)
**1**	Solvent free	NaOH	0.3	70	3	80
**2**	CH_3_CN	NaOH	0.3	Reflux	4	45
**3**	EtOH	NaOH	0.3	Reflux	1	78
**4**	H_2_O	NaOH	0.3	70	1	98
**5**	EtOH:H_2_O	NaOH	0.3	70	1	85
**6**	DMSO	NaOH	0.3	70	2	55
**7**	H_2_O:DMSO	NaOH	0.3	70	2	60
**8**	CH_2_Cl_2_	NaOH	0.3	Reflux	1	50
**9**	PEG-400	NaOH	0.3	70	1	92
**10**	H_2_O	Et_3_N	0.3	70	1	70
**11**	H_2_O	KF	0.3	70	1	45
**12**	H_2_O	NaF	0.3	70	1	65
**13**	H_2_O	NaOH	-	70	24	Trace
**14**	H_2_O	NaOH	0.1	70	1	80
**15**	H_2_O	NaOH	0.2	70	1	90
**16**	H_2_O	NaOH	0.4	70	1	98
**17**	H_2_O	NaOH	0.3	50	1	73
**18**	H_2_O	NaOH	0.3	60	1	87
**19**	H_2_O	NaOH	0.3	80	1	98
**20**	H_2_O	NaOH	0.3	90	1	95

a Isolated yield.

b Reaction conditions: Iodobenzene (1 mmol) and triethoxyphenylsilane (1.5 mmol), and base (2 mmol), Fe_3_O_4_@CNF ∼ ImSBL ∼ Co., and Solvent (3 ml), temperature.

While in the absence of the catalyst did not show significant performance (Table 2, entry 13). The reaction was performed in different amounts of temperature (Table 2, entry 17–20), where the low temperature continued with lower efficiency (Table 2, entry 17). According to the observed results, the optimal conditions for this reaction are: Fe_3_O_4_@CNF ∼ ImSBL ∼ Co. catalyst (0.3 mol%), NaOH (2 mmol) as base in the water at 70^o^C conditions (Table 2, entry 4). After optimizing the reaction conditions, the catalytic effectiveness of Fe_3_O_4_@CNF ∼ ImSBL ∼ Co. MNPs was perused in the Hiyama C-C cross-coupling reactions of a wide range of mercantile available aryl halides with triethoxyphenylsilane as phenylation source. The results are listed in (Table 3) in which the target products were afforded in moderate to excellent yields. The experimental results show that various ortho-, meta-, and para-substituted aryl halides; including, aryl iodide, aryl bromides and aryl chlorides having both electron-withdrawing and electron-donating groups such as NO_2_, CN, Cl and OCH_3_ produced their corresponding derivatives in good to excellent yields. However, it is worth mentioning that the reaction time of the aryl halides with electron-withdrawing groups on the aromatic ring was longer than aryl halides with electron-donating groups. Due to the fact that the aryl halides are electrophilic partners in the Hyiama reaction, they have been activated by electron-donating groups in the para positions, in the oxidative addition step as compared to those with electron-withdrawing groups. Moreover, I, Br, and Cl leaving groups in aryl halides delivered little difference yields, which increasing output was as the order of I > Br > Cl. This effective reaction efficiency between Chloride, Bromide, and iodide leaving groups on aryl halides was another influence of imidazolium moiety in the catalyst according to the proposed mechanism (refer to Scheme 4). Another important point for the Hyiama catalysed by Fe_3_O_4_@CNF ∼ ImSBL ∼ Co. was its high selectivity so that no homo-coupling or any other side-coupling product was observed.

RETRACTED

**TABLE 3:** Recycling activity of the Fe_3_O_4_@CNF ∼ ImSBL ∼ Co. NPs.

Entry	Product	X	R	Time (h)	TON	TOF	E factor	Yield (%)^a^
**1**	3 a	I	H	1	327	327	1.9	98
**2**	3 b	I	4-NO_2_	2	317	158	1.4	95
**3**	3 d	I	4-OMe	3	300	100	1.6	90
**4**	3 c	I	4-Cl	1.5	317	211	1.5	95
**5**	3 e	Br	H	2.5	317	127	1.6	95
**6**	3 f	Br	4-NO_2_	3	323	108	1.2	97
**7**	3 h	Br	4-OMe	5	283	57	1.3	85
**8**	3 g	Br	4-Cl	3	300	100	1.3	90
**9**	3 i	Cl	H	3	300	100	1.3	90
**10**	3 j	Cl	4-NO_2_	2.5	300	120	1.6	90
**11**	3 k	Cl	4-OMe	6	283	47	1.1	85
**12**	3 l	Cl	4-CN	3	267	89	1.1	80

a Isolated yield.

b Reaction conditions: catalyst (0.3 mol%), Aryl halide (1 mmol), triethoxyphenylsilane (1.5 mmol), NaOH (2 mmol).

**SCHEME 4:** A plausible mechanism for the Suzuki–Miyaura and Hiyama cross-coupling reactions catalyzed by the Fe_3_O_4_@CNF ∼ ImSBL ∼ Co.

After receiving the effective results from the Hiyama reaction in the next part of this research project, the binding reaction leading to the aryl compounds through the Suzuki-Miyavra cross-reaction was considered. For this purpose, the coupling of iodobenzene with phenylboronic acid was selected as the model reaction to optimize the reaction conditions. Afterward, the effect of various parameters including solvent, base, amount of the catalyst, and temperature on the reaction efficiency was studied (Table 4). Initially, the effect of the solvent on the outcome of the reaction was studied (Table 4, entry 1–9). It was found that water is the most effective solvent for this type of coupling reaction. (Table 4, entry 4). Then, the effect of the base was examined (Table 4, entry 10–12), the results revealed that the highest yield of the coupling product was obtained in the presence of K_2_CO_3_ as base at 80°C (Table 4, entry 4). In step next, different amounts of the catalyst on the outcome of the reaction was investigated (Table 4, entry 13–16). Among the various catalyst loadings 0.3 mol% of the catalyst on the basis of Co. was selected as the most effective amount (Table 4, entry 4). Meanwhile, in the absence of the catalyst, the reaction didn’t proceed at all even after 24 h (Table 4, entry 13). Eventually, the effect of temperature was examined (Table 4, entry 17–20), the results revealed that the highest yield of the coupling product was obtained at 80°C. Considering the optimized reaction conditions, we studied the overall benefit of our new catalytic system in the Suzuki–Miyaura reaction some aryl halides with phenylboronic acid (Table 5). Different substituted aryl halides were coupled too high to excellent Phenylboronic acid in water at 80°C (Tables 4A–L). It should be noted that electron-withdrawing groups and electron donor groups on aryl halides increase or decrease efficiency. In addition, I, Br, and Cl leaving groups in aryl halides gave a small yield, which increased production I > Br > Cl, respectively. This yields an effective reaction between chloride, bromide, and iodide. Leaving groups on aryl halides was another effect. Another important point for Suzuki–Miyaura, which is catalyzed by Fe_3_O_4_@CNF ∼ ImSBL ∼ Co., is its high choice so that no coupling (normal glazer reaction) or any other by-products were observed.

RETRACTED

**TABLE 4:** Optimization of the reaction conditions for the C-C cross coupling of iodobenzene with t phenylboronic acid.

Entry	Solvent	Base	Catalyst (mol%)	Temp. (^o^C)	Time (h)	Yield^a^ (%)
1	Solvent free	K_2_CO_3_	0.3	80	3	85
2	CH_3_CN	K_2_CO_3_	0.3	Reflux	4	47
3	EtOH	K_2_CO_3_	0.3	Reflux	1	75
4	H_2_O	K_2_CO_3_	0.3	80	1	95
5	EtOH:H_2_O	K_2_CO_3_	0.3	80	1	84
6	DMSO	K_2_CO_3_	0.3	80	2	60
7	H_2_O:DMSO	K_2_CO_3_	0.3	80	2	55
8	CH_2_Cl_2_	K_2_CO_3_	0.3	Reflux	1	45
9	PEG-400	K_2_CO_3_	0.3	80	1	90
10	H_2_O	Et_3_N	0.3	80	1	70
11	H_2_O	NaOH	0.3	80	1	40
12	H_2_O	KOH	0.3	80	1	60
13	H_2_O	K_2_CO_3_	-	80	24	Trace
14	H_2_O	K_2_CO_3_	0.1	80	1	80
15	H_2_O	K_2_CO_3_	0.2	80	1	90
16	H_2_O	K_2_CO_3_	0.4	80	1	92
17	H_2_O	K_2_CO_3_	0.3	50	1	75
18	H_2_O	K_2_CO_3_	0.3	60	1	85
19	H_2_O	K_2_CO_3_	0.3	70	1	90
20	H_2_O	K_2_CO_3_	0.3	90	1	95

a Isolated yield.

b Reaction conditions: Iodobenzene (1 mmol) and phenylboronic acid (1 mmol), and base (2 mmol), Fe_3_O_4_@CNF ∼ ImSBL ∼ Co., and Solvent (3 ml), temperature.

**TABLE 5:** Suzuki–Miyaura reaction of aryl halides with phenylboronic acid catalyzed by Fe_3_O_4_@CNF ∼ ImSBL ∼ Co. in water.

Entry	Product	X	R	Time (h)	TON	TOF	E factor	Yield^a^ (%)
1	3 a	I	H	1	317	317	1.1	95
2	3 b	I	4-NO_2_	2	310	155	0.92	93
3	3 d	I	4-OMe	2	300	150	0.95	90
4	3 c	I	4-Cl	1	300	300	0.93	90
5	3 e	Br	H	1.5	307	205	0.83	92
6	3 f	Br	4-NO_2_	2	327	164	0.64	98
7	3 h	Br	4-OMe	3.5	290	83	0.69	87
8	3 g	Br	4-Cl	2	300	150	0.68	90
9	3 i	Cl	H	3	307	102	0.26	92
10	3 j	Cl	4-NO_2_	1.5	300	200	0.42	90
11	3 k	Cl	4-OMe	7	290	41	0.45	87
12	3 l	Cl	4-CN	2.5	300	120	0.46	90

a Isolated yield.

b Reaction conditions: catalyst (0.3 mol%), Aryl halide (1 mmol), phenylboronic acid (1 mmol), K_2_CO_3_ (2 mmol).

Again, a variety of aryl halides were served in order to coupling with phenylboronic acid under optimum conditions. A same result was found for the effect of leaving groups and electron-withdrawing groups on efficiency of the coupling products (Table 4). Based on the results, aryl halides with electron-withdrawing groups show higher efficiency in these reactions. Iodine as a good leaving group showed a successfully C-C transformation. As shown in Table 4, the exchange of the aryl halides did not have a clear steric effect on the reaction. The cobalt-catalysed Suzuki–Miyaura reaction mechanism comprises the multi-general steps shown in Scheme 4. In addition, leaving groups on aryl halides had other effects on the progress of the reactions. I, Br, and Cl leaving groups in aryl halides gave a small yield, which increased production I > Br > Cl, respectively. This yields an effective reaction between chloride, bromide, and iodide. The presence of imidazole in the catalyst plays an important role in promoting the reactions according to the reaction conditions.

RETRACTED

Because the reaction medium is a water solvent, organic molecules approach the surface of the catalyst to escape water, and the polar nature of the ionic part of the catalyst, which is adjacent to the cobalt ion, causes the components to come together and helping to accelerate the Hiyama and Suzuki–Miyaura cross-coupling reactions. To demonstrate the synergistic effects of different catalyst components (Scheme 3) as well as their performance, including Fe_3_O_4_@CNF, Fe_3_O_4_@CNF-imidazole, SBL ∼ Co. and Co. (OAc) _2_, some analogs were prepared and tested as a catalyst in the Hiyama and Suzuki model reactions.

**SCHEME 3:** Chemical structure of Fe_3_O_4_@CNF, Fe_3_O_4_@CNF ∼ Im, and SBL ∼ Co. as three analogues of the main catalyst.

The results showed that in the model reaction of cobalt salts no detectable products were obtained. (Figure 11). Fe_3_O_4_@CNF nanoparticles did not exhibit any catalytic effect as the core and magnetic substrate. On the other hand, homolog Fe_3_O_4_@CNF ∼ Im, which only had imidazole coordinated by the core-shell Fe_3_O_4_@CNF, produced higher yields than Fe_3_O_4_@CNF under identical conditions (Figure 11, Fe_3_O_4_@CNF ∼ Im: 60–55%). In the next step, the synergistic effect of the encoded metal and ligand was investigated. Homolog SBL-Co of the main catalyst yielded 68 and 75% of the Hiyama and Suzuki–Miyaura coupling product. In the end, to demonstrate the effect of cobalt and ionic liquid group on the model reactions, the reactions were performed in the presence of both Fe_3_O_4_@CNF ∼ Im and SBL ∼ Co. (simultaneously: Fe_3_O_4_@CNF ∼ ImSBL ∼ Co. in the water solvent. As expected, the presence of ionic liquids with metal increases the catalytic properties. For this purpose, as shown in Scheme 3, the Fe_3_O_4_@CNF ∼ ImSBL ∼ Co. catalyst was made so that the imidazole was first coordinated by SBL ∼ Co. groups, and at a later time, cobalt ion was coordinated between the two-dentate Schiff base ligands. The results showed that Fe_3_O_4_@CNF ∼ ImSBL ∼ Co. catalyst provides 95 and 98% yield over 1 h for the model Hiyama and Suzuki–Miyaura reactions under optimum conditions. To demonstrate the strength of the catalyst and its reuse, recycling was performed on the catalyst in the Hiyama and Suzuki–Miyaura reactions.

RETRACTED

**FIGURE 11:** Comparison of the performance of catalysts with each other. ^a^ Fe_3_O_4_@CNF; ^b^ Fe_3_O_4_@CNF ∼ Im; ^c^ SBL-Co (0.3 mol%); ^d^ Co(OAc)_2_.4H_2_O (0.3 mol%); ^e^ Fe_3_O_4_@CNF ∼ ImSBL ∼ Co. (0.3 mol%). Reaction conditions: Hiyama: iodobenzene (1 mmol) and triethoxyphenylsilane (1.5 mmol), and NaOH (2 mmol), Cat (except noted, 0.006 g), and H_2_O (3 ml), T = 70^o^C. Reaction conditions: Suzuki–Miyaura: iodobenzene (1 mmol) and phenylboronic acid (1 mmol), and K_2_CO_3_ (2 mmol), Cat (except noted, 0.006 g), and H_2_O (3 ml), T = 80^o^C.

Recycling of heterogeneous catalysts is especially important for commercial applications. Therefore, the possibility of repeated use of Fe_3_O_4_@CNF ∼ ImSBL ∼ Co. in the reactions described in the previous steps is important. Therefore, the reusability of the Fe_3_O_4_@CNF ∼ ImSBL ∼ Co. di-nuclear catalyst was studied under optimized conditions for the Hiyama and Suzuki–Miyaura model reactions. As exhibited in Figure 12, the catalyst was recovered and reused for at least six consecutive runs. The yield of Hiyama reached 88% and Suzuki–Miyaura reached 87% for the 6th run, which means that only a 10 and 8% drop in efficiency was observed compared to the corresponding fresh catalyst (98 and 95%). Also, to show durability and structure of the catalyst, the recovered catalyst after 6th run was subjected to some analyses. Also, metal leaching of the catalyst was measured in each cycle.

**FIGURE 12:** Recyclability and leaching studies of the Fe_3_O_4_@CNF ∼ ImSBL ∼ Co. nanocatalyst.

As shown in Figure 12, a few leaching was observed for Fe_3_O_4_@CNF ∼ ImSBL ∼ Co., whereas only 3% for Hiyama reaction and 3% for Suzuki–Miyaura reaction metal leaching was observed after the 6th run. Moreover, ICP analysis of the catalyst for each heavy metal demonstrated an insignificant change in their weight percentage than the corresponding fresh values: Fe 46.38, Si 2.23, Co. 7.6 w%. These results demonstrated insignificant changes in the percentages of the heavy metals and confirm the durability of the catalyst during recycling. Finally, in order to ensure the structure of the recovered catalyst was retained, we studied it after the 6th run over the Hiyama model reaction of iodobenzene and triethoxyphenylsilane under the obtained premium conditions by some analyses (Figure 13). FTIR and XRD analysis of the recovered catalyst corroborated that the structure of the catalyst remained completely intact during recycling (Figure 13). The FE-SEM image showed that the nanoparticles were still approximately spherical in shape even after the 6th cycle. It was worth noting that the nanocatalyst showed good magnetism by VSM (Figure 13).

RETRACTED

**FIGURE 13:** **(A)** Fourier-transform infrared, **(B)** vibrating-sample magnetometry curves (I = before ruse and II = after reuse), **(C)** X-ray diffraction spectra, and **(D)** FE-SEM for fresh (green) catalyst after six recovery steps for the Hiyama reaction.

## Comparative Study

The last part of our studies, to demonstrate the profit of Fe_3_O_4_@CNF ∼ ImSBL ∼ Co. as a heterogeneous catalyst in Suzuki–Miyaura reaction, our resultant and reaction conditions were compared with those of some reported Co. catalysts in the Suzuki–Miyaura reaction (Table 6). As depicted in Table 5, the Fe_3_O_4_@CNF ∼ ImSBL ∼ Co. is the most efficient catalyst for the C-C coupling reactions of aryl iodides, bromides, and chlorides. Especially, most of the reported methods toil from the absence of commonness for the coupling reactions of aryl chlorides. In addition, the reported synthetic paths have some limitations, such as requiring high temperature or large amounts of the catalyst, and most importantly, the use of organic solvents. Promising results obtained in the presence of the Fe_3_O_4_@CNF ∼ ImSBL ∼ Co. should be ascribed to the water dispersibility of the catalyst. Because water is dispersible, it increases the possibility of contact between the catalyst and the reactants, and as a result, the stability of the catalyst is greatly increased.

**TABLE 6:** Comparison of catalytic activity of Fe_3_O_4_@CNF ∼ ImSBL ∼ Co. catalyst with some reported cobalt catalysts for Suzuki–Miyaura cross-coupling reactions.

Entry [ref]	Catalyst (mol%)	Reaction conditions	X	Time (h)	Yield (%)
1[Kumar and Bhat (2017)]	Cobalt pincer complex (0.5)	CH_3_CN, 80°C	Cl	16	68
			Br	16	40–83
			I	16	71–90
2[Rasheeda et al. (2017)]	Cobalt Schiff-base complex^a^ (2)	CH_3_CN, 80°C	Br	16	40–83^b^
			I	16	58–79^b^
3[Saroja and Bhat (2019)]	CoASGO^c^ (0.32)	EtOH, 80°C	Cl	24	18, 23
			Br	12–24	45–89
			I	8	97.1^b^
4[Ansari et al. (2018)]	Cobalt salen complex^d^ (2)	Refluxing 1,4-dioxane	Br	8	35–80
			I	8	68.85
5[Akhlaghinia et al. (2017)]	Fe_3_O_4_@Boehmite-NH_2_-Co (0.33)	H_2_O, 80°C	Cl	2–9	15–65
			Br	0.5–4	50–95
			I	3	60–98
6[Sharma et al. (2019)]	Co.@ GO/Fe_3_O_4_/L-dopa^d^ (1.84)	H_2_O, 100°C	Cl	4–8	62–72
			Br	5–7	65–82
7^This Work^	Fe_3_O_4_@CNF ∼ ImSBL ∼ Co. (0.3)	H_2_O, 70°C	Cl Br	1.5–3	87–92
			I	1.5–3.5	87–98
				1–2	90–95

a A complex between 4-aminoacetophenone, salicylaldehyde and cobalt acetate.

b GC yield.

c Cobalt Schiff-base immobilized on graphene nanosheet.

d A salen of *o*-phenylenediamine and salicylaldehyde.

e L-3,4-Dihydroxyphenylalanine.

RETRACTED

### Mechanism Studies

It is worth to note that a few papers, which suggest a mechanism for the cobalt-catalysed cross-coupling reactions, are available in the literature (Ghosh et al., 2016; Mohammadinezhad and Akhlaghinia, 2017; Ansari et al., 2017; Kumar et al., 2017; Sharma et al., 2019), Following these reports, an appropriate mechanism for the biaryl derivatives synthesis reaction catalysed by Fe_3_O_4_@CNF ∼ ImSBL ∼ Co. was proposed (See Scheme 4). Firstly, the reaction was supposed to be started by *in-situ* reduction of Co(II) in the catalyst to Co(I) or Co(0) species under basic conditions (Kumar and Bhat, 2017). Then with the addition of aryl halides are interceded to reduced Co. types by cobalt aryl (I) was formed. Phenylboronic acid, on the other hand, interferes with imidazolium ions to produce (II) the product, which then enters the catalytic cycle. Eventually, the C-C bond provides two six-membered rings, and the biaryl product is produced (III), and the catalyst re-enters the catalytic cycle. Hiyama reaction mechanism is similar to the Suzuki–Miyaura reaction mechanism.

## Conclusion

In continuing the research, a catalytic system with unique properties was designed, synthesize and reported. In summary, we have developed a binucler catalyst on the magnetic cellulose nanofibre with schiff base-Co (denoted as Fe_3_O_4_@CNF ∼ ImSBL ∼ Co.) with high catalytic activity as superparamagnetic nature catalyst, non-toxicity, low cost, easy separation of the catalyst from the reaction mixture by external magnetic field and stability for efficient Hiyama and Suzuki–Miyaura cross-coupling reactions. All the reactions were performed *via* a green process, moderate to high, and excellent conversions in some cases, were achieved for all of entries which this method used is very efficient and useful and tolerates large functional groups with high efficiency. In this way, the catalyst made in the reaction conditions is stable and active for six consecutive times, which is of great importance in terms of environmental issues. We characterized the catalyst from various aspects analyses. The highlight point of the work was of the heterogeneous ionic liquid part, it seems this catalytic system is bi-functional that its imidazole moiety as an ionic liquid shows a useful performance. Because the reaction medium is a water solvent, organic molecules approach the surface of the catalyst to escape the water, and the polar nature of the ionic part of the catalyst, which is adjacent to the cobalt ion, causes the components to come together and helping to accelerate the Hiyama and Suzuki–Miyaura cross-coupling reactions, while on the other hand, the Co(II) complex moiety catalyses the reaction. This methodology is proposed as an affordable alternative to the previous use of noble metal catalysts, especially Pd-based catalytic systems.

RETRACTED

## Data Availability

The datasets presented in this study can be found in online repositories. The names of the repository/repositories and accession number(s) can be found in the article/Supplementary Material.
